# The Exosomes Containing LINC00461 Originated from Multiple Myeloma Inhibit the Osteoblast Differentiation of Bone Mesenchymal Stem Cells via Sponging miR-324-3p

**DOI:** 10.1155/2022/3282860

**Published:** 2022-01-25

**Authors:** Yang Wu, Zhemei Zhang, Jing Wu, Jinxia Hou, Guosheng Ding

**Affiliations:** Clinical Laboratory Center, Gansu Provincial Hospital, Lanzhou 730000, Gansu, China

## Abstract

Multiple myeloma is one of the hematological malignancies and inhibited osteoblast differentiation of bone marrow mesenchymal stem cells (BM-MSCs) which has been proved as a major complication of the patients with multiple myeloma. However, the pathomechanism of symptom remains unclear. Besides, several studies have indicated that LINC00461 plays an important role in the progression of multiple tumors. Hence, this study attempted to reveal the role of LINC00461 in the osteoblast differentiation of MSCs. In this study, the expression level of LINC00461 in the exosomes of multiple myeloma cells was measured, and BM-MSCs were cultured with the exosomes to observe the change of cellular phenotype. Moreover, downstream target of LINC00461 was searched and verified with dual-luciferase reporter assay, and the activation of the Wnt/*β*-catenin pathway was also observed by Western blot. The results showed that the isolated BMSCs exhibited special biomarkers of MSCs. LINC00461 was significantly upregulated in the exosomes originated multiple myeloma cells, and increased LINC00461 significantly impeded the osteoblast differentiation of MSCs. Moreover, LINC00461 could significantly suppress the activation of the Wnt/*β*-catenin pathway in MSCs. In conclusion, this study suggested that LINC00461 in exosomes of multiple myeloma could reduce the activity of the Wnt/*β*-catenin pathway to inhibit the osteoblast differentiation of BM-MSCs via targeting miR-324-3p.

## 1. Introduction

Multiple myeloma is the most dangerous malignant hematological diseases with high morbidity. Statically, more than 100000 people have been diagnosed with multiple myeloma, and approximately 2% cancer-related death in the world is caused by this disease each year [1, 2]. At present, even with the current therapeutic strategies, including radiotherapy, chemotherapy, and drug intervention, the prognosis of the patients with multiple myeloma remains unsatisfactory [3]. According the recent study, the 5-year survival rate of the multiple myeloma is less than 40% [4]. Therefore, investigating more effective intervention techniques for multiple myeloma are urgent.

The failure of osteoblast differentiation is a major reason causing the bone-related complications of the patients with multiple myeloma, such as osteoporosis and osteodynia, which is also related with the malignant progression and of multiple myeloma [5]. The osteoblast differentiation of human mesenchymal stromal cells (hMSCs) serves as an important role in maintaining the stability of skeletal internal environment [6]. Recently, increasing studies have indicated that multiple myeloma cells can remarkably inhibit the differentiation of MSCs, and the intervention on osteoblast differentiation of MSCs has also been confirmed as a promising strategy for alleviating the poor prognosis of the patients with multiple myeloma [7, 8]. Several studies have indicated the aberrant expression of some noncoding RNAs, such as long noncoding RNA (lncRNA) and micro-RNA (miRNA). lncRNA consist of almost 200 ribonucleic acids, and miRNA contains approximately 22 ribonucleic acids [8, 9]. lncRNA and miRNA involve the progression of cellular development and differentiation, and lager studies in recent ten years have illustrated that those aberrant noncoding RNAs involve the formation and development of multiple diseases [8, 10].

LINC00461 has been confirmed as a tumor promoter involving the malignant progressions of many cancer cells [11]. However, few studies have revealed the functions of LINC00461 in multiple myeloma. Thus, this study attempted to investigate the role of LINC00461 in multiple myeloma cells and then reveal the molecular mechanism of LINC00461 on osteoblast differentiation of BM-MSCs.

## 2. Materials and Methods

### 2.1. BM-MSCs Isolation and Osteogenic Differentiation

This study was approved by the hospital ethic committee, and the human-related experiments were performed following the Declaration of Helsinki protocol. The primary CD 138^+^ BM cells were isolated from mononuclear cells of the patients and normal donors. The BM-MSCs obtained from the patients and health donors were cultured with Dulbecco's modified Eagle medium (DMEM) with 20% fetal bovine serum (FBS).

After cell attachment, BM-MSCs were cultured with the osteogenic induction medium (full culture medium containing 10^−2^ M *β*-sodium glycerophosphate, 50 mg/mL L-ascorbic acid, and 10^−7^ M dexamethasone) to induce the progression of osteoblast differentiation. After culture for 21 days, BM-MSCs were strained with alizarin red S (Beyotime), and then, the osteoblast mineralization in three random microscopic regions was imaged and quantified with Image-Pro Plus 6.0 software. Finally, the relative mineralized regions were calculated.

### 2.2. Cell Culture and Translation

Human normal plasma cell line (nPCs) and human myeloma cell lines including H929 and U266 cell lines purchased from Tongpai Biotechnology Co., Ltd (Shanghai, China), and the cells were cultured with the 1640 medium containing 10% FBS. All cells were cultured in an incubator with 5% CO_2_ and 37°C. The cells subculture was performed when the confluence of the cells was at 90%.

The cell transfection was performed when cellular confluence was at 70%. In brief, 4 *μ*g of DNA or 100 pmol RNA was incubated with 250 *μ*l serum-free mediums for 5 min and then was mixed and incubated with isometric serum-free containing 10 *μ*l Lipofectamine 2000 at 25°C for 20 min. Finally, the mixtures were added into each well, and the cells were further incubated for 24 hours.

### 2.3. Exosomes Isolation

U266 cells were cultured with FBS-free 1640 medium, and the culture medium was collected and centrifuged at 800 g for 5 min, followed by 3000 g for 10 min and 10000 g for 60. After that, total exosome isolation reagent (Cat#: 4478359; Thermo Fisher Scientific) was used for isolation of exosomes from the supernatants. Afterward, exosomes were harvested from the pellets and resuspended in PBS. Then, 0.22 *μ*m pore size polyvinylidene difluoride (PVDF) membrane filters (Cat#: GVWP04700; Millipore Sigma) were used to filter any remaining cells or debris. The concentration of exosome was quantified through the BCA kit.

### 2.4. Cells Differentiation and Observation

The MSCs were cultured and induced with osteogenic differentiation medium, including alpha-minimum essential medium containing 10% FBS, 2 mM L-glutamine, 100 mM dexamethasone, 0.2 mM L-ascorbic acid, and 10 mM *β*-glycerophosphate. The osteogenic differentiation of BM-MSC cells were observed after alizarin red staining. In brief, the MSCs were fixed with 1% formaldehyde for 15 min after inducing with osteogenic differentiation medium, and then, the cells were rinsed with double distilled water. After that, the cells were stained with 2% alizarin red S solution (pH = 4.2, Shanghai Zeye Biotechnology Co., Ltd, Shanghai, China) for 10 min. Finally, after rinsing with double distilled water for three times, the cells were imaged and then quantified with decalcification solution at 405 nm.

### 2.5. qRT-PCR

For RNA extraction, the total RNAs of the cells were isolated with TRIzol reagent. The total RNAs were transcribed as cDNA by a PrimeScript® RT reagent Kit (Thermo Fisher, Massachusetts, the USA). The reaction system including primers, cDNA, dNTPs, and Taq DNA polymerase were prepared according the instruction of the qRT-PCR kit (Sigma-Aldrich, Missouri, USA). After that, qRT-PCR was performed according to the following program: denaturation at 95°C for 3 min, followed by amplification for 40 cycles at 95°C for 12 s and at 53°C for 40s and 70°C for 30s. The relative levels of miRNA or mRNA were calculated with the 2^−(ΔΔCt)^ method. The sequences of the primers are given in Table 1.

### 2.6. Western Blot

The total proteins of the cells were extracted with RIPA buffer on the ice, and then, the concentration of the extracts was measured with the BCA kit. The protein was added with loading buffer and then boiled at 100°C for 5 min. After that, 30 *μ*L of the symbol was separated by SDS-polyacrylamide gel electrophoresis (SDS-PAGE), and then, the proteins in the gels were transferred on the polyvinylidene difluoride membranes by the wet transfer method. The membranes were blocked with 5% fat-free milk at 4°C for 2 hours and then were incubated with the related primary antibodies at 4°C overnight. Subsequently, the membranes were washed with TBST for three times, and then, the membranes were incubated with the second antibodies. Finally, the expressions of the related proteins were observed with a chemiluminescence detection system.

### 2.7. Dual-Luciferase Reporter Gene Assay

The binding sites of LINC00461 and miR-324-3p were obtained from the NCBI database (https://www.ncbi.nlm.nih.gov/) and used for synthetizing the mutant sequences of LINC00461. The mutant type and wild type of LINC00461 were, respectively, cotransfected with miR-324-3p mimics or the miR-NC into HEK-293T for 48 hours. After that, a dual-luciferase reporter assay system was used to observe the luciferase activity of HEK-293T.

### 2.8. Data Analysis

The experiments in this study were performed 3 times, independently. The data analysis was performed with SPSS 20.0 with the chi-squared test or ANOVA with Tukey's post hoc-test and then were graphed with GraphPad Prism 8.0. Moreover, *P* < 0.05 meant that the statistically significance existed in two groups.

## 3. Results

### 3.1. LINC00461 Was Upregulated in the Exosomes of Multiple Myeloma Cells

To analyze the role of LINC00461 in multiple myeloma cells, the expression levels of LINC00461 in cells and pathological symbol were measured with qRT-PCR. The result showed that LINC00461 was significantly upregulated in multiple myeloma cells, compared with the normal cells (Figure 1(a), *P* < 0.01). Moreover, the increased LINC00461 was also found in the exosomes originated from multiple myeloma cells (Figure 1(b), *P* < 0.01). Those observations suggested that LINC00461 may involve the progression of multiple myeloma and was abundant in the exosomes of multiple myeloma cells.

### 3.2. The Exosomes of Multiple Myeloma Cells and LINC00461 Inhibited the Osteoblast Differentiation of MSCs

To investigate the mechanism of multiple myeloma cells on blocking the osteoblast differentiation of MSCs, the exosomes originated from MSCs were used to culture MSCs cells. The results showed that compared with normal MSCs, the expression levels of RUNX2 and ALP were downregulated, significantly (Figures 2(a)–2(c), *P* < 0.01). Moreover, compared with the cells transfected with negative control of LINC00461, MSCs transfected with LINC00461-expressed vectors exhibited poor progression of osteoblast differentiation (Figure 2(d), *P* < 0.01). Those observations suggested that LINC00461 was the main substance in the exosomes, which could restrain the osteoblast differentiation of MSCs.

### 3.3. MiR-324-3p Was a Downstream Target of LINC00461

To reveal the regulation mechanism of LINC00461 in development of multiple myeloma, the downstream targets of LINC00461 were searched and matched with TargetScan, an online database. The results showed that miR-324-3p was a potential downstream target of LINC00461 (Figure 3(a), *P* < 0.01). The binding effect of LINC00461 and miR-324-3p was verified by dual-luciferase reporter assay, and the results showed that LINC00461 could directly target 3′-UTR of miR-324-3p. Moreover, the expression level of mi-485-5p was also detected with qRT-PCR. The results showed that miR-324-3p was significantly downregulated in MSCs after transfecting with LINC00461-expressed vectors (Figure 3(b), *P* < 0.05). Those observations suggested that miR-324-3p was a downstream target of LINC00461, and miR-324-3p also involved in the progression of multiple myeloma.

### 3.4. MiR-324-3p Reversed the Effect of LINC00461 on the Osteoblast Differentiation of the MSCs

To further confirm whether miR-324-3p is involved in the regulation of LINC00461 on osteoblast differentiation of MSCs and proosteocytic cells, the miR-324-3p inhibitors and miR-324-3p mimics were cotransfected into cells. The results showed that compared with LINC00461-negative cells, the levels of RUNX2 and ALP in MSCs cotransfected with LINC00461-expressed vectors and miR-324-3p mimics were reversed, partly (Figures 4(a)–4(c), *P* < 0.01). Moreover, the inhibited osteoblast differentiation of MSCs treated with exosomes of multiple myeloma cells was remarkably reversed after transfecting with miR-324-3p mimics (Figure 4(d), *P* < 0.01). Those observations supported that LINC00461 could inhibit the osteoblast differentiation of MSCs and proosteocytic cells via targeting miR-324-3p.

### 3.5. LINC00461 Reduced the Activity of Wnt/*β*-Catenin Pathways via Targeting miR-324-3p

To delve the regulation mechanism of LINC00461 in the progression of multiple myeloma, the activities of the Wnt/*β*-catenin pathway were observed by Western blot. The study showed that Wnt and *β*-catenin were remarkably downregulated in MSCs after transfecting with LINC00461-expressed vectors (Figure 5, *P* < 0.01). Moreover, to further investigate whether miR-324-3p was involved in the regulation of miR-324-3p on multiple myeloma cells, the LINC00461-expressed vectors and miR-324-3p mimics were cotransfected into MSCs, and Western blot showed that the effect of LINC00461 on multiple myeloma could be reversed by increased miR-324-3p (Figure 5, *P* < 0.01). Those observations suggested that LINC00461 could inactivate the Wnt/*β*-catenin pathway via targeting miR-324-3p.

## 4. Discussion

Multiple myeloma is still a malignant plasma cell disorder, which seriously threatens the health of people, and several studies have indicated that the suppressed osteoblast differentiation of the MSCs induced by multiple myeloma can promote the progression of bone-related disease [12]. lncRNA and miRNA involve in the life activities of cells, and the aberrant expression of those noncoding RNA may serve as a key biomarker and drug target reference for clinical treatment [13]. This study proved the relationship of LINC00461 and multiple myeloma and the revealed the regulation mechanism of LINC00461 on osteoblast differentiation of the MSCs.

lncRNA disorder is closely related with the progression of multiple myeloma [14]. In this study, it was found that LINC00461 was significantly upregulated in the multiple myeloma cells and their exosomes. Several studies have indicated that LINC0046 plays a tumor promoter role in some cancer cells and involves the multiple malignant behaviors of the tumor cell, including drug resistance, proliferation, and migration [15]. Qu et al. confirmed that LINC00461 is extremely upregulated in the rectal cancer cells and could decrease the sensitivity of tumor cells on cisplatin via mediating the miR-593-5p/CCND1 pathway [11]. The failure of osteoblast differentiation induced by multiple myeloma has been identified as a major reason leading the poor prognosis of the patients [16]. Increased RUNX2 and ALP have been confirmed as the biomarker events for the differentiation of BMSCs [17]. This study also found that the exosomes originated from multiple myeloma cells or upregulation of LINC00461 could obviously inhibit expression of RUNX2 and ALP. Exosomes, the nanometre-sized membranous vesicles with a diameter of about 30–100 nm, are secreted through the endocytic pathway [18]. The exosomes containing some cancerogenic factors can be released by tumor cells and then may promote angiogenesis and stromal remodelling. Liu et al. indicated that the exosomes derived from multiple myeloma could effectively block the differentiation of BMSCs [19]. Therefore, those study suggested that LINC00461 silence induced the differentiation of osteoblast.

lncRNAs are characterized by regulating the cellular activities via serving as a molecular sponge to specially combine with the related mRNAs and miRNAs. Dong et al. indicated that LINC00461 promotes the proliferation and migration via regulating miR-30a-5p/integrin *β*3 axis [20]. The studies have indicated that miR-324-3p serves as a tumor inhibitor to impede the progression of some cancer cells. Zhao et al. observed that miR-324-3p was remarkably downregulated in thyroid cancer, and increased miR-324-3p could effectively block the progression of hemangioma via targeting PDRG1 [21]. In this study, it was found that LINC00461 could directly target the 3′-UTR of miR-324-3p. It was also found that miR-324-5p was downregulated in the MSCs cells transfected with LINC00461-expressed vectors, and miR-324-3p could partly reverse the effect of LINC00461 on the osteoblast differentiation of MSCs. Kocijan et al. [22] confirmed that the expression of miR-324-3p was correlated with formation and development of the patients with postmenopausal osteoporosis. Moreover, the study also confirmed that miR-324-3p upregulation could partly reverse the effect of LINC00461 on osteoblast differentiation of MSCs. Those proofs suggested that LINC00461 in the exosomes originated from multiple myeloma cells could impede the osteoblast differentiation of MSCs via targeting miR-324-5p.

Cell differentiation involves the changes of multiple signaling pathways, and increasing studies have indicated that the activation of the Wnt/*β*-catenin pathway is responsible for osteoblast differentiation [23]. The study has indicated that the antagonists produced and secreted by multiple myeloma cells may block the progression of osteoblast differentiation via inactivating the Wnt/*β*-catenin pathway in MSCs [24]. In this study, it was found that the expression levels of Wnt and *β*-catenin in MSCs were obviously downregulated after treating with the exosomes of multiple myeloma cells and LINC00461-expressed vectors, suggesting that LINC00461 regulates the osteoblast differentiation of MSCs via inactivating the Wnt/*β*-catenin pathway. Moreover, it was also observed that increased miR-324-3pcould partly reverse the inactivated Wnt/*β*-catenin pathway [25]. Razny et al. indicated that miR-324-3p was significantly downregulated in the progression of osteoblast differentiation, which may be related with the activation of the Wnt/*β*-catenin pathway [26]. Thus, those proofs suggested that LINC00461 could inactivate the Wnt/*β*-catenin pathway to suppress the osteoblast differentiation of MSCs via targeting miR-324-3p.

## Figures and Tables

**Figure 1:** LINC00461 significantly upregulated in the multiple myeloma cells and their exosomes. (a) The relative expression level of LINC00461 in normal and multiple myeloma cell lines. (b) The relative expression level of LINC00461 in the exosomes originated from nPCs and U266.

**Figure 2:** LINC00461 inhibits the osteoblast differentiation of MSCs. (a)–(c) The relative expression levels of RUNX2 and ALP measured with Western blot. (d) The osteoblast differentiation of MSCs observed by alizarin red staining.

**Figure 3:** MiR-324-3p was a target of LINC00461, and miR-324-3p was related with osteoblast differentiation of MSCs. (a) The binding effect of LINC00461 and miR-324-3p observed by dual-luciferase assay. (b) Increased miR-324-3p observed in MSCs during the osteoblast differentiation.

**Figure 4:** LINC00461 inhibits the osteoblast differentiation of MSCs via targeting miR-324-3p. (a)–(c) The relative expression levels of RUNX2 and ALP measured with Western blot. (d) The osteoblast differentiation of MSCs observed by alizarin red staining.

**Figure 5:** LINC00461 inhibits Wnt/*β*-catenin via targeting miR-324-3p. (a)–(c) The expression levels of Wnt and *β*-catenin measured by Western blot.

**Table 1:** Primer sequences of LINC00461, miR-324-3p, and U6.

Name of primer	Sequences
LINC00461-F	5′-GCGTGGACTACTCTGATG-3′
LINC00461-R	5′-CCAAGTGCTTACTGTCT-3′
miR-324-3p-F	5′-ATTAGCCCACTGCCCCAGGT-3′
miR-324-3p-R	5′-CCCACTGCCCCAGGTGCTGCTGG-3′
U6-F	5′-CTCGCTTCGGCAGCACA-3′
U6-R	5′-AACGCTTCACGAATTTGCGT-3′

## Data Availability

The data used to support the findings of this study are available from the corresponding author upon request.
